The article "Role of Glial Cell-Derived Oxidative Stress in Blood-Brain Barrier Damage after Acute Ischemic Stroke" was retracted in 2024. Reasons: signs of a paper mill; compromised peer review; unreliable results or conclusions.

# Role of Glial Cell-Derived Oxidative Stress in Blood-Brain Barrier Damage after Acute Ischemic Stroke

**DOI:** 10.1155/2022/7762078

**Published:** 2022-09-02

**Authors:** Xiaoyan Hu, Yanping Wang, Weihong Du, Li-Jun Liang, Wei Wang, Xinchun Jin

**Affiliations:** ^1^Beijing Key Laboratory of Cancer Invasion and Metastasis Research, Department of Histology and Embryology, School of Basic Medical Sciences, Advanced Innovation Center for Human Brain Protection, Capital Medical University, Beijing 100069, China; ^2^Department of Neurology, The Second Hospital of Jiaxing City, Jiaxing, 314000 Zhejiang, China; ^3^Children's Hospital of Shanxi Province, Taiyuan, Shanxi Province, China; ^4^Department of Physiology and Pathophysiology, School of Basic Medical Sciences, Capital Medical University, Beijing 100069, China

## Abstract

The integrity of the blood-brain barrier (BBB) is mainly maintained by endothelial cells and basement membrane and could be regulated by pericytes, neurons, and glial cells including astrocytes, microglia, oligodendrocytes (OLs), and oligodendrocyte progenitor cells (OPCs). BBB damage is the main pathological basis of hemorrhage transformation (HT) and vasogenic edema after stroke. In addition, BBB damage-induced HT and vasogenic edema will aggravate the secondary brain tissue damage. Of note, after reperfusion, oxidative stress-initiated cascade plays a critical role in the BBB damage after acute ischemic stroke (AIS). Although endothelial cells are the target of oxidative stress, the role of glial cell-derived oxidative stress in BBB damage after AIS also should receive more attention. In the current review, we first introduce the physiology and pathophysiology of the BBB, then we summarize the possible mechanisms related to BBB damage after AIS. We aim to characterize the role of glial cell-derived oxidative stress in BBB damage after AIS and discuss the role of oxidative stress in astrocytes, microglia cells and oligodendrocytes in after AIS, respectively.

## 1. Introduction

Stroke, a common acute cerebrovascular disease, accounts for approximately 9% of all death worldwide and is the second leading cause of death in addition to cardiovascular disease [1]. Stroke is prevalent in the middle-aged and elderly population and is receiving increasing attention in an increasingly ageing society [2]. Stroke is characterized by high morbidity, disability, and mortality rates and can be divided into hemorrhagic stroke and ischemic stroke, the latter of which accounts for 87% of stroke patients [3]. For treatment of acute ischemic stroke (AIS), tissue plasminogen activator (tPA) is the only thrombolytic drug approved by the Food and Drug Administration (FDA), but its clinical use is limited by a strict time window (within 4.5 hours of stroke onset), the high risk of cerebral hemorrhage transformation (HT) after thrombolysis, and high death rate following HT [4]. Because of these limitations, thrombolytic therapy is given to only 3% of patients suffering from AIS [5].

The article "Role of Glial Cell-Derived Oxidative Stress in Blood-Brain Barrier Damage after Acute Ischemic Stroke" was retracted in 2024. Reasons: signs of a paper mill; compromised peer review; unreliable results or conclusions.

After the onset of cerebral ischemia, a series of pathological events are triggered, including energy depletion, excitotoxicity, oxidative stress, inflammation, BBB disruption, and cell death [6]. HT caused by BBB damage aggravate the secondary brain tissue damage [7]. In addition, there is evidence that 25-30% of ischemic stroke survivors develop immediate or delayed vascular cognitive impairment (VCI) or vascular dementia (VaD) [8, 9]. It is therefore crucial to investigate the mechanisms underlying BBB damage after AIS and develop the strategies to protect BBB integrity to reduce secondary brain damage.

The BBB prevents harmful neurotoxic plasma components, blood cells, and pathogens from entering the brain. In addition, BBB also regulates the transport of molecules in and out of the central nervous system (CNS) to maintain its normal function. BBB integrity is mainly maintained by the tight junction proteins (TJPs) between endothelial cells and the basement membrane covering the endothelial cell surface. Meanwhile, BBB integrity is also regulated by other cells in the CNS, such as glial cells [9, 10]. In recent years, glial cells have gradually attracted interests of scientists and doctors. They not only support cells in the CNS but also participates in the progression of related neuropathology such as ischemia-reperfusion injury. The new perspective regards microglia, astrocytes, OLs, and OPCs as exciting therapeutic targets for the treatment of AIS [6, 11]. However, the specific roles of glial cells as well as the underlying mechanisms after AIS need further investigation.

As mentioned above, the current treatments for AIS are intravenous thrombolysis and endovascular mechanical thrombectomy which would induce recanalization. However, reperfusion results in the production of large amounts of reactive oxygen species (ROS), which are responsible for most of the ischemia-reperfusion injury, resulting in brain tissue damage. In addition, oxidative stress can lead to apoptosis, autophagy, and necrosis of brain cells [12]. Therefore, it is crucial to fully understand the mechanisms by which oxidative stress is generated after AIS. Because of the high oxygen consumption, previous research and reviews addressing oxidative stress-induced damage have mainly focused on the neurons within the brain. This review is aimed at summarizing how glial cells influence both the integrity of the BBB and the development of oxidative stress after stroke, providing new ideas for future stroke treatment from the perspective of glial cells.

The article "Role of Glial Cell-Derived Oxidative Stress in Blood-Brain Barrier Damage after Acute Ischemic Stroke" was retracted in 2024. Reasons: signs of a paper mill; compromised peer review; unreliable results or conclusions.

## 2. Physiology and Pathophysiology of the Blood-Brain Barrier (BBB)

### 2.1. Endothelial Cells and Basement Membrane in the BBB

BBB is a highly selective semipermeable membrane barrier that separates blood circulating in the brain from brain tissue. The BBB is a highly differentiated endothelial cell structure of the neurovascular system, consisting mainly of brain microvascular endothelial cells (BMECs), basement membrane (BM), astrocytes end feet surrounding the microvasculature, and pericytes (Figure 1(a)) [13].

Endothelial cells (ECs), joined by tight junctions and adherent junctions, form the first barrier of the BBB for selective passage of intra- and extravascular substances [14–16]. In addition, ECs produce and release various vascular regulatory factors such as endothelin, nitric oxide (NO), and vascular endothelial growth factor (VEGF) to regulate brain microcirculation [17].

The basement membrane (BM) that surrounds ECs forms a second barrier to the BBB. The BM is a complex layer of extracellular matrix proteins that provides support for epithelial and endothelial cells, separating these cells from the brain tissue, thereby contributing to the development, formation, and maintenance of the BBB [18, 19].

### 2.2. Regulation of BBB Integrity by Astrocytes, Pericytes, and Neurons

Astrocytes play an important role in maintaining the integrity of the BBB. It has been shown that the brain microvasculature can maintain its integrity in the presence of massive astrocyte loss, suggesting that astrocytes are not directly involved in the maintaining the integrity of the BBB [20]. Astrocytes are primarily involved in maintaining the integrity of the BBB through releasing certain active substances, in particular growth factors such as VEGF and glial cell-derived neurotrophic factor. In addition, astrocytes are also able to influence the integrity of the BBB by regulating the expression of intracellular cyclic adenosine monophosphate (cAMP) and other proteins [17].

Pericytes are flat, undifferentiated, contractile connective tissue cells that surround the capillary wall [21]. Pericytes synthesize and secrete albumin as an important step in maintaining the integrity of the BBB [22]. During stroke, pericytes migrate away from the vasculature, thereby contributing to increased BBB permeability [23, 24].

Neurons are the most basic structural and functional units of the nervous system, which play the role of connecting and integrating input information and outputting information [25]. BBB regulation in response to neural activity is possibly a direct action of neurotransmitters on cells of the BBB. Of note, acute increases in neural activity in adult animals have also been implicated in changes in BBB function [26], and aberrantly, high neural activity has also been correlated with BBB high permeability [27]. In addition, Lacoste et al. showed that neuronal activity modulates vascular plasticity in the postnatal brain. Moreover, deprivation of sensory input from the barrel cortex of mice, either by surgical deafferent or by genetic inhibition of neurotransmitter release, results in reduced blood vessel density after birth [9]. Neuronal regulation of the BBB and neurovascular coupling has been reviewed by Kaplan et al. [28].

The article "Role of Glial Cell-Derived Oxidative Stress in Blood-Brain Barrier Damage after Acute Ischemic Stroke" was retracted in 2024. Reasons: signs of a paper mill; compromised peer review; unreliable results or conclusions.

### 2.3. Regulation of BBB Integrity by Microglia, Oligodendrocytes (OLs), and Oligodendrocyte Progenitor Cells (OPCs)

Microglia, the resident macrophages of the CNS, numbering 10-15% of the total cell population of the brain, are extremely responsive to changes in the CNS microenvironment and are involved in the homeostatic regulation of the CNS [29]. Microglia are brain microvessel-associated cells. They alter tight junction assembly and BBB permeability by releasing vasoactive substances and cytokines [30, 31]. Normally, microglia are in a quiescent state. Under pathological condition, microglia are activated to either M1 or M2 type [32]. M1 microglia have proinflammatory and prokilling functions. In contrast, M2 microglia are involved in immune regulation, control of inflammatory mechanisms, and repair of damage resolution [33]. Studies have shown that microglia activation is directly related to BBB integrity [34]. Microglia activation may be triggered by microorganisms (e.g., bacteria and virus) or neurodegenerative diseases such as Alzheimer's disease (AD), Parkinson's disease (PD), or stroke. Microglia activation is one of the earliest events in cerebral ischemic events, occurring within minutes to hours after AIS [6, 35]. Therefore, microglia activity is crucial for prognostic and mechanistic investigation after AIS.

Oligodendrocytes (OLs) are myelinating cells of the CNS derived from oligodendrocyte progenitor cells (OPCs), which are widely distributed in the CNS and account for 5%-8% of glial cells [36]. Abnormal oligodendrocyte function underlies the pathology of a range of diseases including stroke, multiple sclerosis (MS), schizophrenia, and AD [37]. After AIS, the function of OLs is impaired, leading to impaired myelin formation on the surface of neurons, followed by impaired neurological function and brain tissue damage [37]. Recent studies have shown that under physiological or pathological conditions, OLs release extracellular vesicles (EVs) into neurons. EVs carry proteins including myelin-associated proteins, which can modulate BBB integrity by regulating neuronal function and neurovascular coupling [38]. Niu et al. showed that in AD patients, interactions between OLs and vascular are disrupted. This interferes with the integrity of endothelial tight junctions and astrocytes end feet, thereby disrupting the BBB and increasing vascular permeability [39]. When white matter is damaged, inflammation and oxidative stress stimulate the release of large amounts of matrix metalloproteinase 9 (MMP-9) from OLs and OPCs, resulting the disruption of the structure of blood vessels and inhibition of the restoration of the BBB [40].

The article "Role of Glial Cell-Derived Oxidative Stress in Blood-Brain Barrier Damage after Acute Ischemic Stroke" was retracted in 2024. Reasons: signs of a paper mill; compromised peer review; unreliable results or conclusions.

### 2.4. BBB Damage in Neurological Diseases

The crucial role of the BBB impairment in the pathological processes of neurological diseases (VCI, VaD, AD, PD, ischemic stroke, MS, and amyotrophic lateral sclerosis (ALS)) received special attention just for a few years [41, 42]. BBB dysfunction begins in the hippocampus in early stage of AD detected with magnetic resonance imaging, and BBB damage may initiate a range of tissue damage, lead to synaptic and neuronal dysfunction and cognitive impairment, end with AD [43]. Notably, BBB breakdown and vascular dysfunction are hallmarks of AD, and targeting BBB has great translational potential in AD therapy [44].

BBB disruption also plays an important role in the pathogenesis of PD, which is characterized by progressive degeneration of dopaminergic neurons in the substantia nigra (SN) [45]. For example, the expression of TJPs decreased, along with increased vascular permeability and accumulation of oligomeric *α*-syn in activated astrocytes of mice brain [46]. In addition, astrocytic VEGFA has been shown to be an essential mediator in BBB disruption in PD [47]. Of note, BBB dysfunction could be detected in PD patients accompanied by the decrease of the function of P-glycoprotein (P-gp), a special protein in the blood vessels of the brain [48]. Therefore, BBB disruption precedes the loss of numerous dopaminergic neurons in the SN and has been hypothesized to contribute to the progression of PD [49].

BBB disruption after stroke was induced by inflammation-driven injury including oxidative stress, increased production of matrix metalloproteinases (MMP), activation of microglia, and infiltration of peripheral immune cells into ischemic tissues [50]. Aging-related vulnerability of the BBB increases the risk and exacerbates the severity of AIS [51]. The role of BBB in aging and neurodegeneration has been reviewed by Knox et al. [52], and BBB impairment is a cause rather than a consequence in aging-related neurodegenerative diseases [53]. Therefore, treatment that could maintain the integrity of BBB would have important roles in preventing aging-related neurological diseases.

The article "Role of Glial Cell-Derived Oxidative Stress in Blood-Brain Barrier Damage after Acute Ischemic Stroke" was retracted in 2024. Reasons: signs of a paper mill; compromised peer review; unreliable results or conclusions.

## 3. Possible Mechanisms Related to BBB Damage after Acute Ischemic Stroke

### 3.1. BBB Damage Induced by Acute Ischemia

After AIS, thrombolysis with tPA within the time window is the only FDA-approved drug. However, its clinical use is limited because of the risk of BBB damage-related vasogenic edema and HT. Jin et al. found that BBB injury occurred firstly in the striatum and preoptic area within 3 hours of cerebral ischemia. The BBB damage area coincides with the brain sites where HT occurred after tPA thrombolysis [54–56]. The mechanisms have been explored, and several signal pathway was involved, such as rapid MMP-2 secretion-mediated occludin degradation and caveolin-1-mediated claudin-5 redistribution [56, 57], neuronal-astroglial cell interactions [58], NO production, and autophagy activation [59]. The BBB damage after AIS is also associated with the neuronal apoptosis induced by neuregulin receptor degradation protein-1, an E3 ubiquitin ligase [60]. The mechanism of BBB injury after AIS is summarized in Figure 1(b). Notably, clinical trials targeting related signaling pathways after AIS are summarized in Table 1.

### 3.2. BBB Damage Induced by Acute Ischemia and Reperfusion

Current treatment for AIS focus on revascularization. However, once blood flow is restored, a series of ischemia-reperfusion injuries will be induced. These include biochemical events, ionic imbalance, oxidative stress, and inflammation, ultimately leading to cellular necrosis and apoptosis. These processes cause massive ROS production, resulting in oxidative stress injury and ultimately brain tissue damage and impaired neurological functions [12].

#### 3.2.1. Inflammation

Inflammatory stimulation is a key mediator of BBB disruption after AIS. Previous studies have shown that inflammation after AIS is mediated by the proinflammatory factors tumor necrosis factor alpha (TNF-*α*) and interleukin-1*β* (IL-1*β*), which are produced between 2 and 6 h after ischemic injury [61]. In addition, proinflammatory factors induce subsequent migration of adhesion molecules, activated neutrophils, lymphocytes, and monocytes into the brain parenchyma [62, 63]. In particular, infiltration of neutrophils plays a key role in enhancing BBB permeability and worsening stroke prognosis [62, 63]. Adhesion molecules such as intercellular adhesion molecule-1 (ICAM-1) and vascular cellular adhesion molecule-1 (VCAM-1), which are expressed at low levels in the BBB, are significantly increased after AIS [64]. It has been shown that inhibition of adhesion molecules or neutrophil integrin proteins may prevent BBB disruption by reducing the number of neutrophils that enter the brain after AIS [65]. In addition, high expression of proinflammatory factors increases the chance of stroke recurrence [66]. The neuroinflammatory response associated with leukocyte infiltration plays an important role in BBB destruction and HT. Inflammatory factors which are released from the ischemic area attract the leukocytes to cross the BBB and enter the brain [67], and leukocyte infiltration may damage the BBB and cause HT by disrupting microvascular endothelial cells. Notably, injection of matrix metalloproteinase 9 (MMP-9) inhibitors can reduce inflammation and the risk of HT during thrombolysis [68].

The article "Role of Glial Cell-Derived Oxidative Stress in Blood-Brain Barrier Damage after Acute Ischemic Stroke" was retracted in 2024. Reasons: signs of a paper mill; compromised peer review; unreliable results or conclusions.

Brain tissue contains lipids with high amounts of unsaturated fatty acids and high concentrations of iron, which make the brain more susceptible to free radicals [69]. Free radicals are divided into two categories: ROS and reactive nitrogen species (RNS). The accumulation of a large number of free radicals plays a key role in many pathological processes of ischemia-reperfusion. Neuronal nitric oxide synthase (nNOS) mediates the production of large amounts of NO in neurons during ischemia, and NO may inhibit the mitochondrial respiratory chain and also react with superoxide radical anion to form highly active peroxynitrite, which increases brain damage. NO reacts with or transforms important biological compounds to generate ROS such as hydroxyl radicals and RNS [70–72].

#### 3.2.2. Oxidative Stress

After cerebral ischemia-reperfusion, the inflammatory response induces the production of a large number of ROS, which eventually leads to oxidative stress [73]. The source of ROS consists of two main ways (Figure 2): (1) enzymatic (products of the mitochondrial electron transport chain, which is the primary way to generate ROS [74], and (2) nonenzymatic, the process requires the production of ROS in the presence of free iron [75].

ROS in the CNS are mainly produced by astrocytes and microglia. Superoxide, one of the most important ROS in the CNS, is produced by enzymes such as xantine oxidase (XO), nicotinamide adenine dinucleotide phosphate (NADPH), or as a by-product of the respiratory chain [76]. ROS include peroxy radical (HO_2_), hydroxyl radical (OH^−^), superoxide anion (O_2_^−^), hydrogen peroxide (H_2_O_2_), hypochlorous acid, and ozone [12]. The neuronal oxidative stress after AIS is mainly divided into three stages. The first stage occurs immediately after ischemia, during which oxygen glucose deprivation (OGD) induces mitochondrial depolarization and uncoupling of mitochondrial respiratory chain in neurons. Intermediates accumulated in the respiratory chain interact with oxygen to generate ROS [77]. The second stage is between 25 and 35 minutes characterized by hypoglycemia and hypoxia. At this time, the intracellular ATP is depleted, and a large amount of XO is activated. The third stage is the reperfusion stage where the oxygenation level increases, producing a large amount of ROS [78]. ROS can act on the basement membrane and cell membrane to cause damage to basement membrane and endothelial cells, eventually leading to BBB damage [79]. Studies have shown that AIS leads to a large amount of ROS production which could regulate the expression of claudin-5 and occludin in the BBB to increase paracellular solute leakage and decrease BBB integrity [31, 80, 81].

The article "Role of Glial Cell-Derived Oxidative Stress in Blood-Brain Barrier Damage after Acute Ischemic Stroke" was retracted in 2024. Reasons: signs of a paper mill; compromised peer review; unreliable results or conclusions.

## 4. Role of Glial Cell-Derived Oxidative Stress in the BBB Damage after Acute Ischemic Stroke

### 4.1. Astrocytes in Stroke

#### 4.1.1. Oxidative Stress in Astrocytes

Astrocytes are critically involved in maintaining the integrity of the BBB. Under physiological conditions, there are clear and distinct boundaries between resting astrocytes. When mild injury occurs, astrocytes begin to proliferate, with hypertrophy of cell bodies and processes accompanied by upregulated expression of GFAP. When the injury was aggravated, astrocytes proliferated massively, and the expression of GFAP was significantly upregulated. The cell body is markedly enlarged, and there is overlap between the cells [82]. There are three main ways of oxidative stress after astrocytes activation: mitochondria-derived oxidative stress, NADPH-derived oxidative stress, and RNS production (Figure 3) [83]. Disrupted mitochondrial function leads to an increase of ROS in astrocytes, resulting in astrocytes proliferation [83]. There is a significant increase of cytoplasmic Ca^2+^ concentration when astrocytes are exposed to OGD. Ca^2+^ accumulates excessively into the mitochondria via voltage-dependent anion channels (VDAC) and mitochondrial calcium unidirectional transporters (MCU), triggering the activation of the mitochondrial permeability transition pore (MPTP). Upon MPTP activation, small molecules are excreted from the mitochondria without selectivity. The discharge of small molecules leads to the dissipation of mitochondrial membrane potential, which ultimately leads to impaired antioxidant pathways and ROS production [74]. In addition, the physiological function of astrocytes is influenced by NADPH-derived oxidative stress. NOX2 and NOX4 are the most abundantly expressed NOX isoforms of the NADPH oxidase (NOX) family in the CNS. Studies have shown that NOX4 is expressed in astrocytes, and its expression regulates oxidative stress in astrocytes [84, 85]. RNS production is another mode of endogenous oxidative stress in astrocytes. All the three isoforms of NOS that are expressed in the CNS are expressed in astrocytes, Ca^2+^/calmodulin-dependent nNOS, endothelial NOS (eNOS), and Ca^2+^-independent inducible NOS (iNOS). NO produced by activated astrocytes can cause the dysfunction of neuron mitochondrial membrane complexes II, III, and IV [86]. NO can enhance S-nitrosylation of protein disulfide isomerase, followed by superoxide dismutase 1 (SOD1) aggregation in astrocytes and enchanced ischemia-reperfusion injury [87].

The article "Role of Glial Cell-Derived Oxidative Stress in Blood-Brain Barrier Damage after Acute Ischemic Stroke" was retracted in 2024. Reasons: signs of a paper mill; compromised peer review; unreliable results or conclusions.

After AIS, activated astrocytes also have positive effects besides their damaging effects. As an important antioxidant and free radical scavenger, glutathione participates in redox reactions and can combine with peroxides and free radicals to reduce ROS toxicity. Astrocytes are rich in glutathione and enzymes related to glutathione metabolism, which play a key role in reducing oxidative stress toxicity and preventing aggravation of ischemic injury [69, 88–91].

#### 4.1.2. Regulation of BBB Permeability by Astrocytes

Astrocytes play an important role in BBB injury after AIS. Endothelial cells and astrocytes were cocultured to mimic *in vitro* BBB and endothelial cells exposed to 24 h OGD caused astrocytes apoptosis by secreting microvesicles accompanied by increased BBB permeability and degradation of the tight junction proteins occludin and claudin-5 [92]. In addition, after AIS, neurons stimulate VEGF production by astrocytes, leading to degradation of the tight junction proteins occludin and claudin-5 and increased permeability of the BBB [93]. In addition, astrocytes can release MMPs and glutamate. MMPs disrupt endothelial TJPs and some kinds of extracellular matrix [94]. Glutamate activates N-methyl-D-aspartate (NMDA) receptors on endothelial cells, inducing vasodilation and increasing BBB permeability [95, 96]. Indeed, astrocytes also produce NO and increase the permeability of the BBB through the cyclic guanosine monophosphate pathway [97, 98]. Moreover, astrocytes produce ET-1 after AIS, an endogenous long-acting vasoconstrictor which overexpression can increase BBB permeability and aggravate brain injury [99, 100].

Astrocytes can produce some cytokines to maintain BBB function. Astrocytes can produce angiopoietin-1 (Ang-1) and Sonic Hedgehog (SHH) and increase endothelial tight junction protein expression and angiogenesis to protect the BBB [101, 102]. Under ischemic conditions, astrocytes can produce insulin-like growth factor-1 (IGF-1) which could stabilize the microvascular cytoskeleton to maintain normal permeability of the BBB [103, 104]. Taken together, astrocytes have a dual role in regulating BBB permeability. How to regulate the secretion of protective factors by astrocytes and to protect the integrity of the BBB requires further research.

The article "Role of Glial Cell-Derived Oxidative Stress in Blood-Brain Barrier Damage after Acute Ischemic Stroke" was retracted in 2024. Reasons: signs of a paper mill; compromised peer review; unreliable results or conclusions.

### 4.2. Microglia in Stroke

#### 4.2.1. Microglia and Oxidative Stress

After AIS, microglia are firstly activated (Figure 4). 24 h after AIS, microglia activation can be detected in the core and peri-infarct areas of ischemic hemisphere [105, 106]. On one hand, activated microglia produce cytokines and chemokines that promote leukocyte infiltration and aggravate the disruption of the BBB and brain tissue [107]. On the other hand, activated microglia may play a beneficial role by phagocytosing cellular debris and suppressing inflammatory responses [17]. The activated microglia can be defined by the expression of surface markers, Iba1, IB4, F4/80, CD11b, and CD68, and increased CD11b expression could indicate the severity of microglia activation [108]. Activated microglia after AIS are polarized into a proinflammatory M1 phenotype or an anti-inflammatory M2 phenotype that produces immunomodulatory molecules such as cytokines and chemokines. It has been shown that M1 microglia promote secondary brain injury, whereas M2 microglia promote recovery after AIS [109, 110]. Inducible nitric oxide synthase (iNOS) and arginase-1 (Arg1) represent a relatively straightforward set of markers to follow M1 versus M2 phenotypes [111]. Roy et al. showed that stimulation of mouse BV-2 microglia and primary microglia with lipopolysaccharide (LPS) promoted upregulation of CD11b expression. Meanwhile, the elevated CD11b expression in microglia was blocked by antioxidants such as N-acetylcysteine and pyrrolidine dithiocarbamate [112]. Inhibition of ROS prevents the proliferation and activation of microglia [113], suggesting that ROS are involved in microglia activation. Mander et al. reported that the proinflammatory cytokines IL-1*β* or TNF-*α* stimulated microglia proliferation, which could be inhibited by a NADPH oxidase inhibitor oleuropein, suggesting that NADPH oxidase-derived hydrogen peroxide mediated the microglia proliferation after AIS [114]. Microglia NADPH oxidase can be rapidly activated by LPS and interferon-gamma (IFN-*γ*), followed by the expression upregulation of iNOS and NO that are induced by ROS release in rat. NAPDH oxidase inhibitors blocked the upregulation, indicating that NAPDH oxidase is involved in the proinflammatory response of microglia, further supporting that NAPDH oxidase-derived ROS are essential for proinflammatory gene expression in glial cells [115].

The article "Role of Glial Cell-Derived Oxidative Stress in Blood-Brain Barrier Damage after Acute Ischemic Stroke" was retracted in 2024. Reasons: signs of a paper mill; compromised peer review; unreliable results or conclusions.

Studies have shown that nuclear factor erythroid 2-related factor 2 (Nrf2) plays a critical role in promoting the transition of microglia to the M2 phenotype. In a Parkinson's disease model, microglia in Nrf2-deficient mice have an increased M1 and a decreased M2 phenotype [116]. In the presence of ROS, microglia may tend to polarize toward M1 and reduce the activation of M2, thus playing an important role in inflammation. It is important to note that M2 microglia have three subtypes, M2a, M2b, and M2c, which are related to the timing of stimulation [117]. The exact role of these three subtypes of M2 microglia in neurological diseases needs further investigation.

#### 4.2.2. The Role of Microglia in Maintaining the BBB Integrity

It has been shown that loss of microglia increases vascular permeability and cerebral hemorrhage, with detrimental effects on vascular density in a neonatal stroke model. Growing evidence demonstrate that the dual roles of microglia exhibited in BBB damage after AIS may depend on the phenotype of microglia. Microglia/macrophages are activated into a proinflammatory or an anti-inflammatory phenotype when they are stimulated [118–120]. After stroke, proinflammatory cytokines such as IL-1*β*, TNF-*α*, and IL-6 are upregulated in M1-type microglia and disrupt BBB integrity by altering cytoskeletal organization, TJP expression, and MMP production [121]. In addition, M1-type microglia increase brain endothelial cell permeability by NADPH oxidase activation-induced P-glycoprotein dysfunction, which leads to the accumulation of neurotoxic molecules in the brain [122]. Inhibiting microglia activation by minocycline, an inhibitor of inflammation, promotes long-term neurovascular remodeling and neurological recovery after ischemia [123]. On the other hand, the complexity of retinal vasculature is reduced if macrophage-colony stimulating factor is deficit in mice, suggesting a potential role for microglia in angiogenesis [124]. After stroke, microglia aggregate around the vascular system, resulting in vascular disintegration and upregulation of phagocytic CD68 expression in the penumbra [125]. Subsequently, microglia released the proangiogenic factor VEGF, suggesting that microglia can promote cerebral vascular remodeling after ischemic stroke [126]. Since microglia play a dual role after stroke, further study are needed to explore how to activate the microglia into an anti-inflammatory phenotype to promote neural recovery after stroke.

### 4.3. Oligodendrocytes and OPC in Stroke

#### 4.3.1. Oligodendrocytes, OPC, and Oxidative Stress

Oligodendrocytes (OLs), the cells responsible for axon myelin formation in the CNS, are deficit in neurological diseases including multiple sclerosis (MS), schizophrenia, and AD [37]. So far, most of ischemia stroke-related studies focus on gray matter, and the role of white matter has been ignored. Actually, white matter damage accounts for about half of the infarction area after cerebral ischemia [127, 128]. In animal models of stroke, the degree of white matter damage is strongly correlated with the age of the animals. It was shown that juvenile animals are more resistant to cerebral ischemia compared to perinatal and old [129, 130], suggesting that white matter damage mechanisms are associated with age.

The article "Role of Glial Cell-Derived Oxidative Stress in Blood-Brain Barrier Damage after Acute Ischemic Stroke" was retracted in 2024. Reasons: signs of a paper mill; compromised peer review; unreliable results or conclusions.

In the early stages of cerebral ischemia, there is an increase in oxidative stress, especially after reperfusion, which leads to OL damage and consequent demyelination, followed by severe long-term sensorimotor and cognitive deficits [131]. During cerebral ischemia, OLs produce large amounts of superoxide radicals, lipid peroxidation, and iron oxidation (Figure 5) [132]. Pantoni et al. showed that 30 minutes after arterial occlusion, OLs, and astrocytes were significantly swollen and 3 h later, a large number of OLs were fatally injured [133]. OPCs are more vulnerable to stimuli than neurons or astrocytes during early reperfusion after stroke [134]. Delayed treatment with the antioxidant ebselenolide significantly reduced transient ischemia-induced gray and white matter injury and neurological deficits, suggesting that oxidative stress plays an important role in the white matter injury after cerebral ischemia [135].

During ischemia, extracellular levels of the neurotransmitters glutamate and ATP are significantly elevated, which triggers OL injury [136, 137]. Excess neurotransmitters overactivate the receptors and cause damage to OLs through excitotoxicity [138]. Glutamate receptor antagonists partially protect against oligodendrocyte damage and reduce white matter injury [139].

#### 4.3.2. The Role of Oligodendrocytes and OPC on BBB Permeability and Angiogenesis

OLs are involved in the regulation of the integrity of the BBB by interacting with endothelial cells. After stroke, OLs secrete MMP-9 which could accelerate the angiogenic response after white matter injury. Primary OLs treated with the proinflammatory cytokine IL-1*β* induces upregulation and secretion of MMP-9. Tube formation was significantly increased if brain endothelial cells were treated with IL-1*β*-conditioned medium of OLs. MMP inhibitor GM6001 was able to inhibit angiogenesis around the injury zone. It is shown that MMP-9 produced by OLs can promote angiogenesis *in vitro* [140, 141]. OPCs secrete the soluble factor TGF-*β*1 that maintains the integrity of the BBB. In an *in vitro* BBB model, OPC-conditioned medium increased tight junction protein expression and decreased BBB permeability by activating the TGF-*β* receptor-MEK/ERK signaling pathway [142]. In neonatal mouse brain, OPCs attached to brain endothelial cells via basement membrane, indicating that OPCs also play a key role in promoting BBB integrity [143]. In addition, OPCs play an important role in facilitating angiogenesis in the brain. Hypoxia causes OPCs to secrete Wnt7a and Wnt7b, which directly stimulate endothelial cell proliferation and promote angiogenesis [144]. Nogo-A is a membrane protein expressed on the surface of OLs and neurons. It is a growth inhibitory, antiadhesion, and growth cone collapse factor. In the postnatal mouse brain, high expression of Nogo-A inhibits angiogenesis, and decreased expression of Nogo-A increases angiogenesis in vivo [145]. Therefore, OPCs may improve neurological recovery by modulating poststroke angiogenesis which is positively associated with the recovery of neurological function after stroke [146].

The article "Role of Glial Cell-Derived Oxidative Stress in Blood-Brain Barrier Damage after Acute Ischemic Stroke" was retracted in 2024. Reasons: signs of a paper mill; compromised peer review; unreliable results or conclusions.

## 5. Conclusion

There is an urgent need to understand the pathophysiological of mechanisms after AIS and the interactions between the various components of the brain. In this review, we discuss the mechanisms of BBB dysfunction after stroke, in particular, the impact of oxidative stress on the BBB. Subsequently, we discuss the important roles of glial cells such as astrocytes, microglia, OPCs, and OLs in oxidative stress after stroke, as well as their impact on the BBB and angiogenesis. Future studies could explore the specific mechanisms of glial cell-mediated oxidative stress, the functional differences between different glial cell types, and the differential effects of different glial cells on the integrity of BBB, which would be a very promising target for the treatment of AIS.

## 6. Literature Search Criteria

Relevant research articles and reviews before June 2022 were retrieved on PubMed using glia, BBB, oxidative stress, and stroke as keywords. References to included studies were manually screened for 150 articles based on the relevance of the title/abstract to the keywords.

## Figures and Tables

**Figure 1:** Components of blood-brain barrier and the mechanisms underlying BBB damage after acute ischemic stroke. (a) Schematic diagram of the BBB structure and other neural cells in the CNS that interact with the BBB. (b) Molecular mechanisms of BBB disruption in the acute phase of ischemia. (1) VEGF produced by activated astrocyte after stroke acts on neurons and causes occludin degradation between endothelial cells. (2) Dopamine receptor activation elevates endogenous tPA in neurons, which causes occludin degradation. (3) The upregulation of HIF-1*α* in neurons increases the expression of MMP-2 in endothelial cells and leads to the degradation of occludin. (4) Caveolin-1 mediates tPA-induced MMP-9 upregulation in cultured brain microvascular endothelial cells. (5) Nitric oxide interacts with caveolin-1 to facilitate autophagy-lysosome-mediated claudin-5 degradation in endothelial cells.

The article "Role of Glial Cell-Derived Oxidative Stress in Blood-Brain Barrier Damage after Acute Ischemic Stroke" was retracted in 2024. Reasons: signs of a paper mill; compromised peer review; unreliable results or conclusions.

**Figure 2:** The mitochondrial electron transport chain under normal conditions and production of ROS. (a) Physiological conditions, electrons are sequentially transferred on complex I, coenzyme Q, complex III, cytochrome C, and complex IV on the inner mitochondrial membrane and finally produce H_2_O and O_2_. (b) The production process of ROS (red). Under pathological conditions, electrons leave the ETC and directly combine with O_2_ to form super oxide radicals-O_2_^−^. O_2_^−^ can generate H_2_O_2_ under the catalysis of SOD. H_2_O_2_ catalyzes the formation of OH^−^ in the presence of metallic Fe^2+^. On the other hand, there are antioxidative pathways in cells (green). H_2_O_2_ can be reduced to H_2_O under the action of GSH via the pentose phosphate pathway. ETC: electron transport chain; NAD^+^: nicotinamide adenine dinucleotide; FADH_2_: flavin adenine dinucleotide; FAD: flavinadeninedinucleotide; Cyt C: cytochrome C; GPx3: glutathione peroxidase 3; GSH: glutathione; GSSG: oxidized glutathione; GR: glutathione reductase.

**Figure 3:** Schematic illustration of the mechanism by which astrocytes activation disrupts BBB integrity after stroke. (a) Astrocytes activation disrupts BBB integrity after stroke. (b) Activated astrocytes allow a large amount of Ca^2+^ to enter mitochondria through VDAC and MCU to generate O_2_^−^. O_2_^−^ exits mitochondria through MPTP to cause oxidative stress. NOX4 promotes oxidative stress in astrocytes. In addition, NOS in astrocytes catalyzes the production of NO to cause RNS. On the other hand, activated astrocytes secrete VEGF and MMPs causing BBB dysfunction.

**Figure 4:** Schematic representation of the effect of microglia activation on BBB integrity after stroke. Microglia are activated to either M1 or M2 type after stroke. They have different effects on BBB integrity. IL-1*β* and TNF-*α* promote M1 microglia activation. IL-4 and Nrf2 promote M2 microglia activation.

**Figure 5:** Schematic representation of the effects of OLs and OPCs on BBB integrity and angiogenesis after stroke. After stroke, the differentiation of OPCs into OLs is blocked. Oxidative stress in damaged OLs causes neuronal demyelination. High expression of Nogo-A in OLs inhibits angiogenesis. Poststroke oligodendrocytes secrete MMP-9, which accelerates angiogenesis following white matter injury. On the other hand, OPCs secrete Wnt7a and Wnt7b to promote angiogenesis after stroke.

The article "Role of Glial Cell-Derived Oxidative Stress in Blood-Brain Barrier Damage after Acute Ischemic Stroke" was retracted in 2024. Reasons: signs of a paper mill; compromised peer review; unreliable results or conclusions.

**Table 1:** Clinical trials targeting signaling pathways related to blood-brain barrier damage.

Signaling pathways	Reference
Autophagy, IL-1, CREB1, mTOR, BER (base extension repair), interferon, relaxin, RAN, estrogen receptor, gas signaling pathway	[147]
AMPK/mTOR signaling pathway	[148]
RBP4/Lp-PLA2/Netrin-1 signaling pathway	[149]
Zinc as a signaling medium	[150]

## Data Availability

No data were used to support this study.

## Abbreviations

AD: Alzheimer's disease
Ang-1: Angiopoietin-1
AIS: Acute ischemic stroke
Arg1: Arginase-1
BBB: Blood-brain barrier
cAMP: Cyclic adenosine monophosphate
CNS: Central nervous system
Cyt C: Cytochrome C
ETC: Electron transport chain
EVs: Extracellular vesicles
FADH2: Flavin adenine dinucleotide
FAD: Flavin adenine dinucleotide
FDA: Food and Drug Administration
GR: Glutathione reductase
GSH: Glutathione
GSSG: Oxidized glutathione
H2O2: Hydrogen peroxide
HO2-: Peroxy radical
HT: Hemorrhagic transformation
ICAM-1: Intercellular adhesion molecule-1
IGF-1: Insulin-like growth factor-1
IL-1*β*: Interleukin-1*β*
iNOS: Inducible nitric oxide synthase
LPS: Lipopolysaccharide
MCU: Mitochondrial calcium unidirectional transporters
MMP-2: Matrix metalloproteinase 2
MMP-9: Matrix metalloproteinase 9
MPTP: Mitochondrial permeability transition pore
MS: Multiple sclerosis
NAD+: Nicotinamide adenine dinucleotide
NADPH: Nicotinamide adenine dinucleotide phosphate
NO: Nitric oxide
NOX: NADPH oxidase
Nrf2: Nuclear factor erythroid 2-related factor 2
O2-: Superoxide anion
OGD: Oxygen glucose deprivation
OH-: Hydroxyl radical
OLs: Oligodendrocytes
OPCs: Oligodendrocyte progenitor cells
RNS: Reactive nitrogen species
ROS: Reactive oxygen species
SHH: Sonic Hedgehog
SN: Substantia nigra
SOD1: Superoxide dismutase 1
TJPs: Tight junction proteins
TNF-*α*: Tumor necrosis factor alpha
tPA: Tissue plasminogen activator
VCAM-1: Vascular cellular adhesion molecule-1
VCI: Vascular cognitive impairment
VDAC: Voltage-dependent anion channels
VD: Vascular dementia
XO: Xantine oxidase.
